The article "Diagnostic Accuracy of 18F-FDG-PET/CT and 18F-FDG-PET/MRI in Detecting Locoregional Recurrence of HNSCC 12 Weeks after the End of Chemoradiotherapy: Single-Center Experience with PET/MRI" was published in 2022. Journal: Contrast Media Mol Imaging.

# Diagnostic Accuracy of ^18^F-FDG-PET/CT and ^18^F-FDG-PET/MRI in Detecting Locoregional Recurrence of HNSCC 12 Weeks after the End of Chemoradiotherapy: Single-Center Experience with PET/MRI

**DOI:** 10.1155/2022/8676787

**Published:** 2022-08-24

**Authors:** Sarita Murtojärvi, Simona Malaspina, Ilpo Kinnunen, Terhi Tuokkola, Miikka-Juhani Honka, Virva Saunavaara, Tuula Tolvanen, Aleksi Schrey, Jukka Kemppainen

**Affiliations:** ^1^Department of Otorhinolaryngology, Turku University Hospital, Turku, Finland; ^2^Turku PET-Centre, Turku University Hospital, Turku, Finland; ^3^Department of Clinical Physiology and Nuclear Medicine, Turku University Hospital, Turku, Finland; ^4^Department of Medical Physics, Turku University Hospital, Turku, Finland

## Abstract

**Purpose:**

In head and neck squamous cell carcinoma (HNSCC), the early diagnosis and efficient detection of recurrences and/or residual tumor after treatment play a very important role in patient's prognosis. Positron emission tomography (PET) using 2-deoxy-2-^18^F-fluoro-D-glucose (^18^F-FDG) has become an established method for the diagnosis of suspected recurrence in head and neck carcinomas. In particular, integrated PET/MRI imaging that provides optimal soft tissue contrast and less dental implant artifacts compared to PET/CT is an intriguing technique for the follow-up imaging of HNSCC patients. The aim of this study was to evaluate the benefit of PET/MRI compared to PET/CT in post-treatment follow-up imaging of HNSCC patients.

**Methods:**

This retrospective observational cohort study consists of 104 patients from our center with histologically confirmed HNSCC. All patients received chemoradiotherapy (CRT) and underwent ^18^F-FDG-PET/CT (*n* = 52) or ^18^F-FDG-PET/MRI (*n* = 52) scan 12 weeks after the end of treatment. Image analysis was performed by two independent readers according to a five-point Likert scale analysis.

**Results:**

PET/MRI was more sensitive (1.00 vs. 0.77) than PET/CT in the detection of locoregional recurrence. PET/MRI also had better negative (1.00 vs. 0.87) predictive values. AUCs for PET/MRI and PET/CT on patient-based analysis were 0.997 (95% CI 0.989–1.000) and 0.890 (95% CI 0.806–0.974), respectively. The comparison of sensitivity, AUCs, and negative predictive values revealed a statistically significant difference, *p* < 0.05. In PET/CT, false-negative and positive findings were observed in the more advanced disease stages, where PET/MRI performed better. Also, false-negative findings were located in the oropharyngeal, laryngeal, and nasopharyngeal regions, where PET/MRI made no false-negative interpretations.

**Conclusion:**

Based on these results, PET/MRI might be considered the modality of choice in detecting locoregional recurrence in HNSCC patients, especially in the more advanced stages in the oral cavity, larynx, or nasopharynx.

## 1. Introduction

Head and neck squamous cell carcinoma (HNSCC) is the sixth most common cancer worldwide, arising from many different anatomical sites within the oral cavity, nasopharynx, oropharynx, hypopharynx, and larynx. Tobacco use, alcohol consumption, and human papilloma virus (HPV) are the most identified risk factors of HNSCC [1]. Early-stage disease is usually treated with single modality (surgery or radiotherapy), leading to high cure rates. However, locally advanced HNSCC requires multimodality complex treatments, including the combination of radiotherapy with chemotherapy or targeted therapies [2].

Despite the recent progress in treatments, a substantial number of patients experience locoregional and/or systemic failure within the first 3 years of definitive therapy. Patients with early-stage disease show recurrence during follow-up in 10–20% of cases [3], whereas the recurrence rate is up to 50% in patients with locally advanced disease, predominantly in locoregional patterns [4]. Recurrent and/or metastatic HNSCC is associated with poor prognosis, and the median overall survival (OS) is less than one (<1) year [5]. If recurrent disease is diagnosed at advanced stage, it has also major impact on expected survival [6–8]. Therefore, an accurate and early detection of suspected recurrence is crucial in the management of patients with HNSCC to improve survival by increasing the effectiveness of salvage therapy, which is the most effective treatment modality in this setting.

Current ESMO and NCCN guidelines on head and neck SCC recommend imaging of the primary site and neck for locally advanced diseases to assess response to chemoradiotherapy and suspect of recurrence 3 months after the end of treatment, even sooner if alarming new symptoms or abnormalities in clinical examination are found [9]. However, conventional imaging (including contrast-enhanced CT and MRI) has limited ability to distinguish between radiation-induced inflammation, fibrosis, and residual or recurrent diseases.

^18^F-FDG PET/CT is nowadays an established method for the diagnosis of suspected recurrence and for planning treatments such as salvage therapy or lymph node dissection, with a high negative predictive value [10–12]. However, post-treatment follow-up and early detection of recurrence of head and neck HNSCC is still a diagnostic challenge because of surgical and radiation therapy-induced tissue alterations, the variable appearances of recurrent tumors, and physiological and inflammatory conditions that mimic disease activation [13, 14].

The optimal follow-up frequency, total follow-up duration, and screening methods in HNSCC after CRT are not well defined. However, the guidelines highlight the importance of the first two to four years after treatment since approximately 80 to 90 percent of all recurrences after curative-intent treatment occur within this timeframe [9]. In the first year, the follow-up frequency is typically every one to three months; in the second year, once in every two to four months; in years 3 to 5, every four to six months; and after five years, every 12 months [15]. The recent guidelines recommend ^18^F-FDG-PET/CT 3 months after CRT for patients with node-positive disease [9]. One retrospective study showed that ^18^F-FDG-PET/CT scans at regular intervals beginning three to four months after treatment were highly sensitive in detecting locoregional or distant recurrences [16]. Due to tissue inflammation or infection caused by side effects of treatments, it is advisable to wait six weeks after surgery or chemotherapy and 12 weeks after CRT before performing follow-up scans [17]. Higher sensitivity was found in PET scans when performed more than ten weeks after CRT [18]. When PET/CT surveillance 12 weeks after the end of CRT was compared to neck dissection, survival was found to be similar, but surveillance resulted in significantly fewer surgical operations and was more cost-effective [19].

In conventional imaging, MRI is known to be a superior imaging method compared to CT in the head and neck region due to excellent soft-tissue contrast, diffusion-weighted imaging (DWI), and DWI-derived apparent diffusion coefficient (ADC) values, which aid distinguishing likely malignant tissues from benign post-treatment changes or localizing anatomically normal sized lymph node metastases [20]. Moreover, MRI has the ability to detect many anatomically challenging findings like laryngeal cartilage and skull base invasion or perineural disease spread [21]. In recent years, the use of hybrid PET/MRI systems in head and neck malignancies has increased because of the superior soft-tissue contrast and lower occurrence of metallic dental implant artifacts compared to PET/CT imaging. Integrated PET/MRI imaging may constitute an attractive alternative to PET/CT as it may combine in a single session the excellent morphological features of MRI with the increased sensitivity and functional information of PET and may improve the differentiation of tumor recurrence from post-treatment related reactive changes or complications.

Loeffelbein et al. studied in a mixed population of head and neck cancer patients the clinical value of retrospective PET/MRI image fusion compared to side-by-side analysis and single modality use of ^18^FDG-PET and MRI alone. They found that retrospective PET/MRI image fusion was beneficial only in selected cases of recurrent diseases [22]. Many previous studies comparing PET/CT and PET/MRI modalities have been performed also with mixed HNSCC patient populations, where scanning indication included both staging and restaging [23, 24]. For primary staging purposes only, PET/MRI has shown to provide accuracy comparable to PET/CT [25]. There are only a limited number of previous prospective studies that have investigated the feasibility of PET/MRI in restaging and detecting recurrence of head and neck malignancies [26–31]. These articles are listed in more detail in Table 1and discussed in more detail later in the Discussion section. In these studies, the time of the follow-up PET scan varies from 6 months to up to four years or is not stated, and the number of patients included is limited. In early study by Nakamoto et al. in which software-based PET and MRI fusion was used, the authors found that PET/MRI was useful especially in evaluating disease recurrence in HNSCC patients, while diagnostic gain was not obtained when assessing primary tumors [32]. Queiroz et al. investigated PET/MRI compared to contrast enhanced PET/CT in 87 patients with suspected recurrence of head and neck cancer. PET/MRI did not yield higher accuracy, but it helped to detect tumor recurrence, mimicking ^18^F-FDG findings [30].

However, no studies that evaluated the diagnostic accuracy of PET/MRI in the specific time window of 12 weeks after CRT have been performed yet. Since the availability of PET/MRI, our center has started using this modality as an alternative to PET/CT in post-chemoradiation treatment evaluation. However, PET/MRI scan for these patients are more expensive and scanning is more time consuming than routine PET/CT modality. Therefore, the aim of this study was to retrospectively evaluate the possible added value of PET/MRI imaging compared to PET/CT in the detection of disease recurrence 12 weeks after the end of chemoradiation treatment from the perspective of a single-center experience.

## 2. Materials and Methods

### 2.1. Patient Selection

This observational cohort study included a total of 104 patients with HNSCC who were referred for a restaging PET scan at the Turku PET Centre, Turku University Hospital, between February 2014 and May 2017. Patients were consecutively selected according to the following inclusion criteria:

1. Histologically confirmed HNSCC with no distant metastases at the time of diagnosis
2. Treatment with chemoradiotherapy

We consecutively selected 52 patients who underwent ^18^F-FDG-PET/CT and 52 patients who underwent 18F-FDG-PET/MRI 12 weeks (mean ± SD: 12.3 ± 1.4 weeks) after the end of treatment. The PET/MRI cohort and the PET/CT cohort consist of the first 52 patients selected in the first three years after our center started using PET/MRI imaging, meeting the inclusion criteria mentioned above.

### 2.2. Chemoradiotherapy Protocols

Patients were treated with intensity-modulated radiation therapy (IMRT) with concurrent chemotherapy including cisplatin or cetuximab. Doses of radiotherapy to the primary tumor varied from 63 to 70 Gray (Gy), the elective dose to the neck was 50 Gy, and doses to lymph node metastases varied from 60 to 70 Gy. Radiotherapy was given in fractions during a period of six weeks, giving two fractions a day and five fractions a week.

Concurrent chemotherapy consisted of weekly dose of cisplatin 40 mg/m^2^, given one to six times, standard treatment being six weeks. Patients treated with cetuximab received a weekly dose of 250 mg/m^2^ for three to seven times, standard treatment being seven weeks. Two patients received a combination of the two chemotherapies.

### 2.3. Histological Diagnosis

All primary tumors were histologically confirmed and staged according to the American Joint Cancer Committee on Cancer (AJCC) staging manual, 7^th^ edition [33]. Biopsy-proven squamous cell carcinomas of unknown origin in cervical lymph nodes were presumed to be head and neck cancers and were included. HPV detection for all patients was performed on collected primary tumor tissue.

### 2.4. PET/CT and PET/MRI Protocol

PET/CT scans were performed using either a 64-row Discovery D690 or VCT PET/CT system (General Electric Healthcare). PET/CT images were acquired in from the level of the eyebrow to mid thigh with 3 min per bed position. Images were reconstructed with an iterative statistical fully three-dimensional maximum-likelihood ordered-subset expectation maximization (OSEM) algorithm. Data were corrected for dead time, decay, and photon attenuation and were reconstructed to a 128 × 128 matrix. Low-dose ultrafast CT protocol (80 mAs, 120 kV) was used for attenuation correction and anatomic correlation.

PET/MRI scans were performed with a sequential Ingenuity 3T TF PET/MRI system (Philips Healthcare) using a SENSE neurovascular coil. MRI sequences dedicated to the neck area were T2 TSE (cor, sag), T1 TSE (ax, sag), and T1 SPIR (ax). The sequences were focused at the area of primary/recurrence tumor and lymph node regions of the neck. The size of scanning areas was time dependent, but by using all those sequences, it was possible to cover a whole area of the neck (between forehead and medial head of clavicles). T1 SPIR and T1 sag sequences were always scanned with contrast media. T2 sequences provided exact anatomical information from both tumor and lymph node areas. T1 sequences with and without contrast media had an essential role for an evaluation of tumor malignancy.

Subsequently, a Dixon and an MRI-based attenuation correction sequences were acquired from the level of the forehead to the groin level. Attenuation correction procedure was performed using a 3-segment model with differentiation of air, lung, and soft tissue.

PET imaging was performed after MRI sequences. Transaxial field of view was 576 mm. PET images were reconstructed using the default reconstruction algorithm “Blob-OS-TF”, a 3D ordered subset iterative TOF reconstruction technique with 3 iterations and 33 subsets. Using 144 × 144 matrices, the final voxel size was 4 × 4 × 4 mm^3^. All reconstructions included the necessary corrections for image quantification: attenuation, randoms, scatter, dead-time, decay, and detector normalization.

All patients fasted for at least 6 hours before PET examination and had a controlled blood glucose level before the radiotracer injection. The mean ± SD of administered ^18^F-FDG activity was 278 ± 53 (284 ± 55.9 MBq for PET/CT and 273 ± 49.1 MBq for PET/MRI). PET/CT and PET/MRI scans began, respectively, 52 ± 4 min and 53 ± 4 min (mean ± SD) after the radiotracer injection.

### 2.5. Image Analysis and Interpretation

Image analysis was performed using an ADW 4.6 workstation (General Electric Medical Systems).

Two independent readers, a nuclear medicine physician and a radiologist, evaluated the PET/CT and PET/MRI images qualitatively according to a five-point Likert scale analysis (1: definitely negative for recurrence; 2: probably negative; 3: indeterminate; 4: probably positive; and 5: definitely positive) [34]. In discordant cases, a consensus decision between the two physicians was reached. PET scans with a score >3 in the local and/or regional area were considered positive for recurrence.

A semiquantitative analysis using SUVmax was also performed on increased ^18^F-FDG uptake both in positive and negative scans. A comparison of the PET/CT and PET/MRI findings according to tumor location, stage, and HPV status was performed.

All patients received clinical follow-up with routine clinical examination and nasopharyngolaryngoscopy by a head and neck surgeon and cross-sectional imaging if needed, according to ESMO clinical practice guidelines on SCC tumors [9]. Time of follow-up from the completion of CRT treatment was at least two years (24 months) in all patients of both cohorts (mean 36 months; SD 24–60 months). Follow-up period was calculated from the date of CRT treatment completion to the last day of follow-up or death by any cause.

Histopathological sampling or imaging follow-up was considered as a reference standard in recurrence diagnosis. Recurrence beyond 12 months from the end of CRT was presumed independent of PET findings in this study.

### 2.6. Statistical Analysis

Mean ± SD was used to present the descriptive features of variables. True-positive (TP), true-negative (TN), false-positive (FP), and false-negative (FN) rates were calculated in relation to reference standard. Sensitivity, specificity, positive predictive value (PPV), and negative predictive value (NPV) were calculated for both imaging modalities and at the patient and lesion levels. Student's *t*-test was performed to evaluate differences between the two cohorts. Moreover, receiver operating characteristics (ROC) analysis was performed on patient- and lesion-based sensitivity and specificity.

Analyses were performed using SAS software, version 9.4, of the SAS System for Windows (Copyright © 2002–2012 SAS Institute Inc., Cary, NC). Areas under the curve (AUCs) in receiver operating characteristics (ROC) analysis were compared using the package pROC [35] of *R* statistical computing environment (version 4.1.0) [36]. Sensitivity, specificity, and positive and negative predictive values; the number of individuals of different sex; and HPV infection between PET/CT and PET/MRI diagnostic studies were compared using the N-1 chi-square test where expected numbers on the contingency tables were at least 1 or otherwise using the Fisher–Irwin test [37]. Tumor location and stage distribution were compared using the chi-square test. The significance level for this study was set at 0.05.

## 3. Results

Patient characteristics are summarized in Table 2. No statistically significant difference (*t*-test, *p*=>0.1) according to age, sex, AJCC stage, tumor location, and HPV status was observed between the two cohorts. In both groups, oral cavity and oropharynx were the most common tumor locations and more than half of tumors were in advanced (stage IV) stage.

Cisplatin treatment was administered to 45 patients in the PET/CT cohort and 35 patients in the PET/MRI cohort. Three patients in the PET/CT group and 4 patients in the PET/MRI group received 3–7 doses of cetuximab instead of cisplatin. In the PET/MRI group, one patient received a combination of 3 doses of cetuximab and 2 doses of cisplatin, and in the PET/CT group, one patient received 1 dose of cetuximab and 5 doses of cisplatin. 15 patients (3 in the PET/MRI group and 12 in the PET/CT group) did not receive chemotherapy due to poor clinical conditions of the patients or toxicity onset. Primary tumor surgery or elective neck dissection before CRT was performed to 51 patients (26 in the PET/CT group and 25 in the PET/MRI group).

All the patients except for one in the PET/MRI group and one in the PET/CT group received radiotherapy. Doses of radiotherapy to the primary tumor(s) varied from 63 to 70 Gy. 41 patients in the PET/MRI group and 42 patients in the PET/CT group received an elective dose to the neck, and the standard dose was 50 Gy, but the final dose varied from 48 to 56 Gy. 39 patients in the PET/CT group and 34 patients in the PET/MRI group received radiotherapy to the neck lymph node metastases, and the dose varied from 60 to 70 Gy. Radiotherapy was given in fractions during a period of six weeks.

During follow-up, histology verification was available in 13 patients from the PET/CT cohort and 8 from the PET/MRI cohort, while follow-up imaging was performed in the remaining patients. Local recurrence was confirmed according to reference standard in 10 (19%) patients in the PET/CT cohort and in 16 (31%) patients in the PET/MRI cohort. Sensitivity, specificity, PPV, and NPV for both imaging modalities at the patient and lesion level are presented in Table 3. Overall, PET/MRI yielded a better diagnostic performance especially in terms of sensitivity, NPV, and PPV, while maintaining a high specificity. AUCs for PET/MRI and PET/CT on patient-based analysis were 0.97 (95% CI 0.989–1.000) and 0.890 (95% CI 0.806–0.974), respectively (Figure 1), and the comparison of AUCs revealed a statistically significant difference (*p*=0.017).

At the patient level, PET/CT had 10% false-negative results, while with PET/MRI no false-negative results were recorded. False-positive interpretations were made three times (6%) in the PET/CT cohort and once (2%) in the PET/MRI cohort. These were most commonly located in oral cavity diseases, one in the PET/CT group and one in PET/MRI group. The remaining two false-positive interpretations in the PET/CT group were located in the larynx (*n* = 1) and in the nasopharynx (*n* = 1). In the PET/CT cohort, there were 5 false-negative cases (9.6%), in the nasopharynx (*n* = 2), oral cavity (*n* = 1), and larynx (*n* = 2).

According to the tumor location, the oral cavity, nasopharynx, and larynx were the regions where false interpretations were made (Figure 2(a)). In oral cavity HNSCC, FP results occurred in both modalities (one in PET/MRI and one in PET/CT). On the other hand, PET/MRI correctly interpreted all findings in the nasopharynx and larynx regions, compared to PET/CT (FN 5, FP 2). According to the stage, in PET/MRI scans, FP results occurred in patients with stages ≥IVA, whereas in PET/CT examinations, FP and FN findings were found in patients with stages ≥III (Figure 2(b)). HPV-positive patients had a higher percentage of true-negative scans confirmed in the follow-up (100% on PET/MRI and 84% on PET/CT) compared to HPV-negative patients (Figure 2(c)).

Mean SUVmax values for recurrent tumors were 6.4 ± 3.0 for PET/CT and 5.7 ± 2.2 for PET/MRI. In false-positive findings, mean SUVmax was 5.1 ± 0.5 in the PET/CT group and 4.2 ± 1.6 in PET/MRI. True-negative findings showed a mean SUVmax of 3.8 ± 0.9 for PET/CT and 3.7 ± 1 for PET/MRI.

## 4. Discussion

In this observational patient cohort study, the impact of the introduction of PET/MRI in the clinical routine as an alternative to PET/CT in diagnosing recurrent HNSCC at 12 weeks after chemoradiotherapy was evaluated retrospectively. It was observed that, in the PET/MRI cohort, there were fewer number of false-positive and false-negative findings demonstrating a better sensitivity and NPV of this method over PET/CT. Interestingly, this study pointed out that false-positive and negative imaging findings were reported in PET/CT imaging to stage III or higher patients with disease localized in the oral cavity, nasopharynx, or larynx. Patients with such characteristics would seem to be more suitable for PET/MRI imaging. There were no false-negative findings during this retrospective analysis in the PET/MRI cohort, and only one false-positive finding was located in the oral cavity in a stage IV patient; whereas, in the PET/CT cohort, the number of false-positive findings was increasing according to disease stage.

Since MRI imaging is known to be superior to CT in HNSCC imaging, it could be assumed that switching from PET/CT to PET/MRI would gain additional clinical benefits as well. Becker et al. in a prospective study of 74 patients showed that PET/MRI is excellent in the detection and T-staging of local recurrence HNSCC after (chemo)radiotherapy [26]. Schaarschmidt et al., in a prospective study including 18 patients, observed no significant differences in the performance of ^18^F-FDG PET/MR, ^18^F-FDG PET/CT, and MRI in local primary staging and cancer recurrence diagnosis. The follow-up PET time in patients with suspected cancer recurrence was not stated [27]. Kubiessa et al. studied 18 patients of whom 10 had a recurrent HNSCC. The follow-up time varied from six months to up to four years. This prospective study showed that PET/MRI has good diagnostic capability, similar to PET/CT [28]. Partovi et al. showed that ^18^F-FDG-PET/MR imaging and ^18^F-FDG-PET/CT provide comparable results in the detection of regional lymph node and distant metastases. This prospective study had 14 patients, and 9 of them had recurrent diseases [29]. Recent studies had not found a statistically significant difference in the ability of PET/CT and PET/MRI in detecting distant metastases in oropharyngeal and hypopharyngeal squamous cell carcinoma [38, 39].

These previous prospective studies (Table 1) had relatively small cohorts, and the groups were quite heterogeneous. For staging purposes, PET/MRI appeared to be at least similar but not superior to PET/CT in diagnostic performance. Moreover, the time of the PET scan after treatment was mentioned or varied a lot, from 6 months up to four years, which makes it challenging to assess the diagnostic performance in the restaging setting. There were few previous studies where PET/CT and PET/MRI are head-to-head compared in the detection of local recurrence of HNSCC after chemoradiotherapy. Queiroz et al. in a prospective study of 87 patients compared locoregional HNSCC recurrence detection. However, the time of the follow-up PET was not defined. The authors observed only marginal differences in diagnostic accuracy between contrast-enhanced (ce) PET/MRI and cePET/CT modalities, but very significant ones when comparing only ceCT to ceMRI [30]. Thus, despite the anatomical reference playing an important role, the sensitivity of the metabolic information provided by PET imaging is more significant in the detection of possible recurrence. Varoquaux et al. studied the quality of PET images and coregistered anatomic images obtained with PET/MRI, evaluated the detection of focal uptake and SUV, and compared these findings with those of PET/CT in patients with head and neck tumors. This prospective study had 32 HNSCC patients, and the follow-up time was not determined. PET/MRI showed equivalent performance to PET/CT in terms of qualitative results. Comparison of SUVs revealed an excellent correlation for measurements on both modalities, but underestimation of SUVs measured on PET/MRI as compared to PET/CT [31].

As presented in Table 1, in the results of Kubiessa et al., PET/CT and PET/MRI reached comparable good specificity (85.5–89.1% for PET/CT and 81.9–94.5% for PET/MRI) and very good NPV for both combined modalities and no statistically significant differences were found [28]. Also, Queiroz et al. found no statistically significant difference in sensitivity, specificity, NPV, and PPV when comparing PET/CT and PET/MRI [30]. In our results, PET/MRI performed better in diagnostic accuracy, sensitivity, and NPV and the difference was statistically significant (*p* < 0.05). One reason for this could be our more homogenous cohorts and a consistent, shorter follow-up time. Becker et al. studied only PET/MRI and found sensitivity of 97.4%, specificity of 91.7%, NPV of 97.1%, and PPV 92.5% [26], which are quite well in line with our findings.

Underdiagnosis of recurrence with CT and MRI imaging may be related to an underestimation of the extent of submucosal disease spread. A diagnostically challenging recurrence pattern is typically multicentric with widespread foci, which is more difficult to localize within post-therapeutic inflammation and fibrosis [40, 41]. In this kind of situations, the higher sensitivity of ^18^F-FDG-PET imaging might increase the detection of possible recurrence. However, ^18^F-FDG-PET can also be a major source of false-positive findings, especially due to tissue inflammation. It has been shown that MRI fused with PET images is able to specify up to 1/3 of the unclear ^18^F-FDG findings [30, 32].

In the light of the promising data in the literature, in our center it was also thought that PET/MRI would improve diagnostic accuracy and patient management [24, 30, 42]. Therefore, according to the available scanner capacity since 2014, our HNSCC patients have been preferably scanned with PET/MRI instead of PET/CT for follow-up and restaging after chemoradiotherapy.

Altogether 3 false-positive patient interpretations were noted with PET/CT, which accounts 6% of the whole cohort. PET/MRI produced 1 false recurrence suspicions accounting 2% in the cohort. The location of the tumor has a great role in early diagnostics. False-positive findings in PET/CT were located in the oral cavity, nasopharynx, and larynx. In oral cavity HNSSC, false-positive results occurred in both modalities. On the other hand, PET/MRI interpreted correctly all findings in the nasopharynx and larynx regions.

False-positive interpretations with PET/CT were made in one larynx and tonsillar SCC patient with suspicion of lymph node metastasis in neck mandibular angle and suspicion of disease recurrence in one patient with tongue cancer, who had physiological ^18^F-FDG uptake in the tongue muscle. False-positive findings in PET/MRI most likely were related to unspecific/reactive ^18^F-FDG uptake in cricoarytenoid muscles and suspected local disease recurrence in the inflammation area close to the tracheostomy tube. Also, more true negatives were noted in HPV-positive than in HPV-negative HNSCC patients, which is in line with previous studies [43].

PET/MRI did not detect any false-negative findings. In the PET/CT cohort, the false-negative findings were in nasopharyngeal and laryngeal regions and in the oral cavity. False-negative findings were related to anatomically challenging regions. All of these recurrences were initially found in clinical examinations and not in the PET/CT imaging. Two of them, both recurrences of laryngeal HNSCC, were found within the following six months, after the patient developed new alarming symptoms.

It is of interest that PET/CT performed well in disease stages I and II, but all false-negative and positive findings were observed in the more advanced stages, stage III and IV, respectively. Our study suggests that in stage II disease the diagnostic performance of PET/CT and PET/MRI is quite similar, but in the more advanced stages PET/MRI seems to be the preferred modality. This is likely related to the ability of PET/MRI imaging to specify unclear ^18^F-FDG findings like postsurgical ^18^F-FDG uptake in the tongue or assessing regions obscured by dental artifacts in CT [6, 24, 30]. Most CT artifacts are related to dental implants and located in the suprahyoid region, in the oral cavity and oropharynx, while main MRI artifacts are related to movement: swallowing, talking, coughing, or even breathing, and this is noted in the infrahyoid regions [24]. It could be hypothesized that one reason for false interpretations in the more advanced disease stages is increased potential for tumor necrosis, which would lead to less uptake seen on PET scans.

Previous review articles have compared the advantages and disadvantages of PET/CT and PET/MRI. Dental implants, tissue inflammation, or local reaction to radiotherapy can cause disturbance in the diagnostic imaging. Dental implants cause more artifacts in PET/CT imaging. PET/MRI seems to be the modality of choice for the evaluation of the oropharynx and the oral cavity because of a higher incidence of artifacts in PET/CT in this area mainly due to dental implants [30]. In PET/MRI, the radiation dose is smaller, but the imaging is more time-consuming and more expensive. In the complex head and neck region, movement artifact due to swallowing, talking, coughing, or even breathing might be a problem, especially in MRI modalities. There are many MRI sequences to reduce the above-mentioned artifacts, but these are significantly more time-consuming and therefore PET/CT may be more feasible in practice as a whole-body imaging method [24]. In ^18^F-FDG-PET imaging, the physiological ^18^F-FDG uptake in Waldeyer's ring or any other lymphoid tissue and activity in laryngeal muscles or vocal cords must be taken into consideration. Also lungs often have physiological activity and movement artifacts due to breathing. Furthermore, in lung imaging, PET/CT is superior in detecting small lung nodules [44]. The mucous membrane of the head and neck region always has some physiological ^18^F-FDG uptake. This may be hard to separate from superficial tumor tissue. Also, the muscles of the flaps used for reconstruction of the tongue after tumor surgery have altered ^18^F-FDG uptake [45]. In these cases, PET/MRI is superior because of its ability to differentiate soft tissue as well as normal from pathological tissue.

It has been shown that diffusion-weighted imaging might not bring additional benefit to primary tumor staging [24, 46]. Whether this is true to treatment response assessment as well is not known. Kuhn et al. demonstrated that T1w cePET/MR and T2w PET/MR performed significantly better regarding conspicuity of primary tumor lesion assessment than PET/CT. In lymph node metastases assessment, the MRI sequences did not perform significantly better. They concluded that required sequences and imaging protocol might depend on whether imaging is for primary staging, therapy response, or tumor recurrence detection. In some cases, ^18^F-FDG PET imaging acts already like a contrast agent and certain circumstances might not yield clinically relevant additional information; for example, in therapy assessment, reduced MR protocol could be used since PET is the major component for the distinction of responders from nonresponders.

Being an observational cohort study, the main limitation of this study is the inability to directly compare the diagnostic performance or the possible additional value that an imaging method has above another leading to different treatment strategies. However, it is worth mentioning that, in comparison to previous literature, our cohort is among the largest ones and especially the more homogenous. The cohorts are comparable in size, disease localization, stage, patient selection, and follow-up time, which limits the risk for selection bias. There are no previous studies where disease location, stage, and imaging modality have assessed as possible sources of false interpretation, and there are no previous studies where the performance of PET/CT and PET/MRI imaging are evaluated systematically 12 weeks after chemoradiotherapy. Moreover, this study is able to provide preliminary data on the better performance of PET-MRI imaging, which showed fewer false-positive and false-negative findings. Finally, we might also tentatively identify a subpopulation of patients that might have a higher risk for false diagnosis depending on PET modality used. Our study in fact suggests that, in stage III or higher disease localized in the oral cavity, nasopharynx, or larynx, PET/MRI could be the method of choice in diagnosing early recurrence after treatment compared to PET/CT.

However, there are other factors that can limit the use of PET/MRI imaging in clinical practice. First of all, PET/MRI scanner availability is still limited worldwide. Secondly, imaging costs are higher along with longer scanning and reading times compared to PET/CT.

In our university hospital, PET is not used routinely to all primary head and neck cancer patients. MRI is the imaging method of choice for primary staging in newly diagnosed cancer patients. PET/CT is recommended only for high-risk patients to exclude distant metastases and patients with cancer of unknown origin (CUP). PET/MRI is routinely used only for those patients treated with chemoradiotherapy or patients with uncertain findings in conventional imaging. Clinicians and radiologists in the Tumor Board have adapted this methodology with ease since it is easy and convenient to compare diagnostic MRI images with post-treatment PET/MRI images in Tumor Board meetings. Also, clinicians have noted higher diagnostic confidence in clinical reports and less follow-up procedures are needed to assess suspicious ^18^F-FDG uptake as compared to previous PET/CT images. Additional benefit is that PET/MRI causes less radiation exposure to chemoradiotherapy-treated patients than PET/CT imaging.

Based on these initial promising results on retrospective data, a prospective registered clinical trial (Clinicaltrial.gov ID NCT04196985) has been initiated in our center to compare PET/MRI and PET/CT at 12 weeks after the end of CRT in a single cohort of HNSCC patients. This trial will also consider the effect of scanning modality on patient treatment strategies and cost-effectiveness. We aim to further evaluate the diagnostic efficacy of these two imaging modalities to define best clinical patient management, and the results of the trial are largely awaited.

## 5. Conclusion

This observational single-center study suggests that PET/MRI has a better diagnostic performance compared to PET/CT in the early detection of HNSCC recurrence after CRT. Therefore, it might be considered the imaging modality of choice in this setting, with particular benefit in patients with more advanced stage HNSCC in the oral cavity, nasopharynx, and larynx. The costs, feasibility, and prolonged imaging times are the main factors that might limit the use of PET/MRI. Further studies prospectively comparing these modalities and their cost efficiency are needed.

## Figures and Tables

**Figure 1:** (a) Patient- and (b) lesion-based receiver operating characteristics (ROC) analysis for ^18^F-FDG-PET/CT (red line) and ^18^F-FDG-PET/MRI (light blue line) imaging.

**Figure 2:** Number of true/false-positive and true/false-negative findings in ^18^F-FDG-PET/CT and ^18^F-FDG-PET/MRI cohorts according to (a) disease location, (b) stage, and (c) HPV status.

**Table 1:** Previous prospective single-center studies of ^18^F-FDG-PET/MRI in HNSCC recurrence detection.

Authors and publication information	Title	Patients	Comparison method	Recurrence	Time from end of CRT to PET	Sensitivity (PET/MRI/PET/CT)	Specificity (PET/MRI/PET/CT)	PPV (PET/MRI/PET/CT)	NPV (PET/MRI/PET/CT)	
Becker et al., European Radiology, 2018	Local recurrence of squamous cell carcinoma of the head and neck after radio(chemo)therapy: diagnostic performance of FDG-PET/MRI with diffusion-weighted sequences	74	PET/MRI only	Local	15 ± 12 months	97.4	91.7	92.5	97.1	

Schaarschmidt et al., EJNMMI, 2016	Locoregional tumour evaluation of squamous cell carcinoma in the head and neck area: a comparison between MRI, PET/CT and integrated PET/MRI	25 (13 recurrences)	Comparison with integrated PET/MRI	Locoregional	Not considered					

Varoquaux et al., EJNMMI, 2014	Detection and quantification of focal uptake in head and neck tumours: ^18^F-FDG PET/MR versus PET/CT	18	Comparison with sequential PET/MRI	Locoregional	Not considered					

Queiroz et al., EJNMMI, 2014	PET/MRI and PET/CT in follow-up of head and neck cancer patients	87	Trimodality PET/CT/MRI	Locoregional	Not considered	86/96	94/96	86/83	94/94	

Kubiessa et al., EJNMMI, 2014	Initial clinical results of simultaneous ^18^F-FDG PET/MRI in comparison to ^18^F-FDG PET/CT in patients with head and neck cancer	17 (10 recurrences)	Comparison with integrated PET/MRI	Locoregional	6 months-4 years	78–82/78–87	81–94/85–89	65–85/71–75	91–94/90–94	

Partovi et al., American Journal of Neuroradiology, 2014	Qualitative and quantitative performance of 18F-FDG-PET/MRI versus ^18^F-FDG-PET/CT in patients with head and neck cancer	14 (9 recurrences)	Comparison with sequential PET/MRI	Regional + distant	Not considered					

**Table 2:** Comparison of patient and disease characteristics between ^18^F-FDG-PET/CT and ^18^F-FDG-PET/MRI imaging cohorts.

	PET/CT	PET/MRI	Difference
Age (mean, DS)	64 ± 9	64 ± 11	*p*=0.9

Sex			*p*=0.8
Male	37 (71%)	36 (69%)	
Female	15 (29%)	16 (31%)	

Tumor location			*p*=0.8
Nasopharynx	6 (11%)	3 (6%)	
Oral cavity	15 (29%)	18 (35%)	
Oropharynx	18 (37%)	14 (28%)	
Larynx	8 (15%)	12 (23%)	
Hypopharynx	3 (6%)	3 (6%)	
Unknown primary	2 (2%)	2 (2%)	

Stage			*p*=0.5
I	—	—	
II	8 (15%)	10 (19%)	
III	15 (29%)	9 (17%)	
IVA	25 (48%)	30 (58%)	
IVB	4 (8%)	3 (6%)	

HPV			*p*=0.3
Positive	17 (33%)	11 (22%)	
Negative	35 (67%)	41 (78%)	

**Table 3:** Number of true/false-positive (TP/FP) and true/false-negative (TN/FN) observations, sensitivity, specificity, PPV, and NPV of ^18^F-FDG-PET/CT and ^18^F-FDG-PET/MRI imaging.

	PET/CT		PET/MRI	
	Patient-based, *n* = 52	Lesion-based, *n* = 92	Patient-based, *n* = 52	Lesion-based, *n* = 89
TP	10	13	17	20
FP	3	4	1	1
TN	34	66	34	63
FN	5	6	0	3
Sensitivity	0.67	0.68	1^*∗*^	0.87
Specificity	0.92	0.94	0.97	0.98
PPV	0.77	0.76	0.94	0.95
NPV	0.87	0.92	1^*∗*^	0.95

^*∗*^=*P* < 0.05.

## Data Availability

The anonymized patient data used to support the findings of this study are available from the corresponding author upon request.
